This article has been retracted.

# Vitamin a deficiency and sleep disturbances related to autism symptoms in children with autism spectrum disorder: a cross-sectional study

**DOI:** 10.1186/s12887-021-02775-0

**Published:** 2021-07-03

**Authors:** Jing Wen, Ting Yang, Jiang Zhu, Min Guo, Xi Lai, Ting Tang, Li Chen, Jie Chen, Ming Xue, Tingyu Li

**Affiliations:** 1 Children’s Nutrition Research Center, Children’s Hospital of Chongqing Medical University, Chongqing Key Laboratory of Child Nutrition and Health, Chongqing, PR China; 2 Ministry of Education Key Laboratory of Child Development and Disorders, Chongqing, PR China; 3 National Clinical Research Center for Child Health and Disorder, Chongqing, PR China; 4 China International Science and Technology Cooperation Base of Child Development and Critical Disorders, Chongqing, PR China; 5 Department of Neurosciences and Neurology, Rutgers New Jersey Medical School, Newark, NJ USA

**Keywords:** Vitamin a deficiency, Sleep disturbances, Autism spectrum disorder, Autism symptoms

## Abstract

**Background:**

Vitamin A deficiency (VAD) and sleep disturbances have been reported in children with autism spectrum disorder (ASD). The influence of vitamin A (VA) levels on sleep regulation and sleep disturbances in ASD has garnered concern. The present study aimed to characterize the association of VA levels with sleep disturbances in children with ASD.

**Methods:**

This cross-sectional study compared children with ASD (*n* = 856) to typically developing children (TDC; *n* = 316). We used the Children’s Sleep Habits Questionnaire to assess sleep disturbances, Childhood Autism Rating Scale to evaluate the severity of autism symptoms, and Autism Behavior Checklist and Social Responsiveness Scale to assess autism behaviors. Serum VA levels were estimated using high-performance liquid chromatography. Multivariable linear regression and two-way analysis of variance were performed to investigate if VAD was related to sleep disturbances in children with ASD.

**Results:**

Children with ASD had lower serum VA levels and a higher prevalence of sleep disturbances than TDC did. The incidence of VAD in ASD children with sleep disturbances was higher, and the symptoms more severe than those without sleep disturbances and TDC. Interestingly, the interaction between VAD and sleep disturbances was associated with the severity of autism symptoms.

**Conclusion:**

VAD and sleep disturbances are associated with the core symptoms of ASD in children. Regular monitoring of sleep and VA levels may be beneficial for children with ASD.

**Trial registration:**

Chinese Clinical Trial Registry, registration number: ChiCTR-ROC-14005442, registration date: December 9th 2014.

## Background

Autism spectrum disorder (ASD) is a neurodevelopmental disorder characterized by core symptoms including deficits in social communication and interaction, speech and language disorders, as well as restricted, repetitive, and stereotyped behaviors [1]. Individuals with ASD also have high rates of behavioral and/or medical comorbidities [2, 3]. Sleep disturbances, with a reported prevalence of 50–80% in children with ASD [4–6] compared with 25–50% in typically developing children (TDC), have attracted substantial attention recently [7, 8]. The impact of sleep disturbances on worsening of autistic symptoms and impairment of cognitive development and daily functioning has been well recognized [9–14]. As such, treatments for sleep disorders in children with ASD are now a routine part of clinical management [15]. While the underlying mechanisms are not clear, multiple neurodevelopmental, medical, psychosocial, and environmental factors have been hypothesized to cause increased sleep disturbances in children with ASD. Abnormalities in melatonin levels and their secretion patterns and in *Clock* or *Clock*-related genes and their synaptic pathways have been suggested as possible intrinsic contributors [6, 16–18].

Vitamin A (VA) is implicated in a wide spectrum of biological processes involved in neural differentiation, neurite outgrowth, and the regulation of circadian rhythms [19, 20]. Our previous study documented vitamin A deficiency (VAD) in a cohort of children with ASD [21]. However, in that study we did not assess sleep and it is unknown whether the findings would be reproducible in another cohort of children with ASD. Further, it is not known whether there are specific characteristics of VAD and sleep disorders in children with ASD, whether the level of VAD correlates with the severity of sleep disturbances, and whether the presence of both VAD and sleep disorders potentiates the severity of core symptoms in children with ASD. We speculated that during development, VAD may be associated with ASD risk factors and related to more severe autism-related behaviors and sleep disturbances in children. In the present study, we aimed to (1) evaluate the prevalence of VAD in children with ASD with and without sleep disturbances, (2) determine the relationship between VA levels and sleep disturbances, and (3) investigate the potential effect of VAD and sleep disturbances on autism symptoms.

## Methods

### Participants

The present study was conducted between November 2015 and January 2018 at the Children’s Hospital of Chongqing Medical University and the Maternal and Child Health Hospital of Hainan Province, China. This study included children with ASD who visited the hospital or who attended special educational institutions and had not been supplemented with any vitamin recently. Their parents or guardians were explained the aim and methodology of the study, and participants (*n* = 856) were enrolled in the study after the children’s parents or guardians provided the informed consent. The diagnosis of ASD was confirmed by the board-certified psychiatrists specialized in this field based on the criteria of the Diagnostic and Statistical Manual of Mental Disorders, Fifth Edition (DSM-5) [1]. Children with ASD whose autism was secondary to other disorders such as Rett syndrome, attention deficit hyperactivity disorder, mental retardation, and other congenital diseases were excluded. TDC group was recruited from the child health departments of the two hospitals, which was sex ratio and age stratification ratio same as ASD group.

Parents or guardians of TDC consented to psychological and neurological examinations for exclusion of any developmental or nervous system disorders, congenital disease or hereditary disease, recent infection and any doses of supplements in the last 6 months. Parents of all participants signed written informed consent, and participation in this research was voluntary. This study was approved by the Institutional Review Board of the Children’s Hospital, Chongqing Medical University.

### Measures

Sociodemographic characteristics of the participants and the existence of sleep disturbances or a history of psychiatric disorders in the family were assessed by a sociodemographic form that was developed by the authors. Information about sleep was collected for all participants using the CSHQ which is an international standard questionnaire for assessment of children’s sleep. The CSHQ were collected through investigators who had received comprehensive professional training, and the questionnaire introduction and detailed guidance are given to the caregivers of the ASD and TDC. The caregivers filled in the CSHQ according to the sleep behavior over the past week, and investigator controlled the quality of the questionnaire. Although the CSHQ was not developed for children with ASD, it has been widely used to characterize sleep disturbances in this population. The CSHQ is a 45-item questionnaire that was revised to eliminate redundant or ambiguous items, resulting in 33 items, which were used to assess sleep disturbances in children by asking about their sleep behavior over the past week. Based on the frequency of a behavior, items in the questionnaire were answered using a three-point Likert scale: “usually” (5–7 times per week), “sometimes” (2–4 times per week), and “rarely” (0–1 time per week) [22]. The scale assesses sleep behavior in eight dimensions, including bedtime resistance, sleep onset delay, sleep duration, sleep anxiety, night waking, parasomnia, disordered sleep, and daytime sleepiness. Total sleep disturbance score is generated from 33 items, with higher scores indicating greater sleep disturbances. A total score of 41 is considered to be the most sensitive cutoff for identifying overall sleep disturbances for further clinical assessment [22]. Although the CSHQ was not developed for children with ASD, it has been widely used to characterize sleep disturbances in this population. The Chinese version of CSHQ has been psychometrically validated [23–25]. In the current sample, the Cronbach’s Alpha coefficient for CSHQ full scale was 0.79 and for the subscales, it ranged from 0.37 (bedtime resistance) to 0.76 (sleep duration) with a median of 0.67. The questionnaire was completed by the authors of this study by interviewing the caregivers of children.

For children with ASD, symptoms of ASD were assessed with the Childhood Autism Rating Scale (CARS) [26], Autism Behavior Checklist (ABC) [27], and Social Responsiveness Scale (SRS) [28]. The caregivers of the ASD and TDC completed the ABC and SRS scales conducted by in-person interviews between the standardized trained investigators. CARS scales were collected through face-to-face structured interviews with caregivers that were conducted by investigators who had received professional training. The investigators controlled the quality of all scales. The CARS is used to determine the presence and severity of autism. Scores range from 15 to 60, with scores between 30 and 36 indicating mild to moderate autism and scores above 36 indicating severe autism [26]. The ABC is used for the screening and diagnosis of ASD and is applicable for individuals between 8 months and 28 years of age. Scores between 53 and 67 indicate a moderate probability of autism, while scores ≥68 indicate a high probability of ASD [27]. The SRS is an assessment of social ability that is used for individuals aged 4 to 18 years. Higher scores indicate greater social impairment, with raw scores < 65 being considered in the normal range [28].

### Laboratory measurements

Venous blood samples (5 mL) were collected at room temperature (approximately 21 °C) at 8:00 am and centrifuged for 10 min at 3000 rpm. The serum was then processed for estimation of retinol concentration using a high-performance liquid chromatograph apparatus (DGU-20As, Shimadzu Corporation, Kyoto, Japan) (C18, 315 nm) operated by the same operator in the same setting (a dark room). Serum retinol concentrations ≥1.05 μmol/L were defined as VA normal (VAN); < 1.05 μmol/L and ≥ 0.7 μmol/L were defined as marginal VA deficiency (MVAD); and < 0.7 μmol/L were defined as VAD [29].

### Statistical analysis

The statistical analyses were performed using IBM SPSS Statistics, version 22.0 (IBM Corp., Armonk, NY, USA). The Kolmogorov–Smirnov goodness-of-fit test was used to test the distribution of each data set for normality before analysis. Continuous variables are presented as means, when appropriate, and categorical variables are presented as frequencies and percentages. To compare VA levels between the groups, one-way analysis of variance (ANOVA), chi-square test, and Fisher’s exact test were used. A two-way ANOVA was conducted to assess the interaction between sleep disturbances and VA levels. The differences for multiple comparisons were analyzed using the Student–Newman–Keuls (SNK-q) test. Multiple linear regression analysis was used to assess the association of VA level and autism symptoms with sleep disturbances. The odds ratios and 95% confidence intervals (95% CI) were calculated for linear regression analyses and statistical significance was set at *P* < 0.05 for all analyses.

The individual enrollment, group design, and testing are shown in Fig. 1. The clinical trial was registered in the Chinese Clinical Trial Registry (ChiCTR) (registration number: ChiCTR-ROC-14005442; registration date: December 9th 2014).

**Fig. 1:** Flow chart representing the study population

## Results

### Participants

In total, 856 children with ASD (692 males, 164 females, male to female ratio 4.22:1) and 316 age- and sex-matched TDC (253 males, 63 females, male to female ratio 4.02:1) were enrolled in the study. Sex distribution in the two groups was not significantly different (χ^2^ = 0.089, *P* = 0.765) (Table 1). The age of parents (fathers: *P* < 0.001; mothers: *P* = 0.005) was significantly higher in the ASD group than the TDC group, which is consistent with other reports [11, 20, 30, 31].

**Table 1:** Comparison of groups for social background variables

Variable	TDC (*n* = 316)	ASD (*n* = 856)	*P* value
**Sex, % (n)**^a,b^			
Male	80.1 (253/316)	80.8 (692/856)	0.765
Female	19.9 (63/316)	19.2 (164/856)	
**Age (years)**, mean (SD)			
Children	6.43 (0.96)	6.27 (2.80)	0.317
Father	29.93 (5.27)	31.02 (2.39)	< 0.001^***^
Mother	27.98 (4.96)	28.82 (2.78)	0.005^**^
**CSHQ total score**, **% (n)** ^c^	49.68 (157/316)	79.67 (682/856)	< 0.001^***^
**VA levels**, mean (SD)	1.05 (0.13)	0.69 (0.33)	< 0.001^***^

*Abbreviations*: *TDC* Typically developing children, *ASD* Autism spectrum disorder, *SD* Standard deviation, *CSHQ* Childhood Sleep Habit Questionnaire, *VA* vitamin A

^**^P < 0.01, ^***^P < 0.001

^a^Sex ratio of male to female was 4.22:1 in ASD group and 4.02:1 in age- and sex-matched TDC group

^b^Obtained from two-sided t test (ANOVA)

^c^ Individuals in ASD and TDC cohorts in this study were consistent in age (4–10 years) according to Owens et al. [22]

### VA levels and sleep disturbances in individuals with ASD

Significant differences in VA levels and sleep disturbances were found between the ASD and TDC groups (Table 1). The mean serum VA level was significantly lower in the ASD group than the TDC group (mean ± standard deviation: 0.69 ± 0.33 μmol/L vs. 1.05 ± 0.13 μmol/L, respectively, *P* < 0.001). The children with ASD had a significantly higher prevalence of sleep disturbances than TDC based on the defined cutoff score of 41 on the CSHQ (ASD: 79% [682/856 children], TDC: 49% [157/316 children], *P* < 0.001).

We additionally analyzed the relationship of VAD and sleep disturbances in the ASD group. Children with ASD were stratified into two groups based on their CSHQ score relative to the cutoff score (over and below 41). Individuals with sleep disturbances (i.e., CSHQ total score over 41), compared to those without sleep disturbances (i.e., CSHQ total score below 41), had significantly lower VA levels (*P* < 0.001) (Table 2). Interestingly, the children with ASD without sleep disturbances had a mean VA level of 1.04 ± 0.15 μmol/L, which was not significantly different from that of the TDC group (1.05 ± 0.13 μmol/L, *P* = 0.274). Furthermore, we found a correlation between the degree of VAD and the prevalence of sleep disturbances. Among children with ASD without sleep disturbances, none had definitive VAD, two-thirds had MVAD, and one-third had normal VA levels. In contrast, more than 60% of individuals with ASD with sleep disturbances had definitive VAD (Table 2). Moreover, when individuals with sleep disturbances were stratified into groups based on VA levels (i.e., VAN, MVAD, and VAD), those in the VAD group had higher CSHQ scores than those in the MVAD and VAN groups (Table 3).

**Table 2:** Comparison of VA levels and core symptoms in ASD children with and without sleep disturbances

Variable	Without sleep disturbances^a^ (*n* = 174)	With sleep disturbances^a^ (*n* = 682)	*P* value
**VA levels**^b^			
VA levels, mean (SD)	1.04 (0.15)	0.60(0.27)	< 0.001^***^
VAN, % (n)	29.89 (52/174)	16.86 (115/682)	< 0.001^***^
MVAD, % (n)	70.11 (122/174)	22.29 (152/682)	
VAD, % (n)	0 (0/174)	60.85 (415/682)	
**CARS score, % (n)**			
Mild to moderate degree (30–36)	54.60 (95/174)	5.43 (37/682)	< 0.001^***^
Severe degree (37–60)	45.40 (79/174)	94.57 (645/682)	
**ABC total score, mean (SD)**	64.13 (7.77)	99.57 (25.05)	< 0.001^***^
**SRS total score, mean (SD)**	91.55 (15.58)	141.24 (30.06)	< 0.001^***^

*Abbreviations*: *ASD* Autism spectrum disorder, *VA* Vitamin A, *SD* Standard deviation, *CARS* Childhood Autism Rating Scale, *ABC* Autism Behavior Checklist, *SRS* Social Responsiveness Scale, *CSHQ* Childhood Sleep Habit Questionnaire

^***^P < 0.001

^a^The individuals with total CSHQ scores below 41 were classified as without sleep disturbances; those with over 41 were classified as with sleep disturbances [22]

^b^Serum retinol concentrations ≥1.05 μmol/L were defined as Vitamin A Normal (VAN); < 1.05 μmol/L and ≥ 0.7 μmol/L were defined as Marginal Vitamin A Deficiency (MVAD); < 0.7 μmol/L were defined as Vitamin A Deficiency (VAD) [29]

**Table 3:** Comparison of the CSHQ, CARS, ABC, and SRS scores in ASD children with sleep disturbances stratified by different VA levels

Variable	Sleep disturbances + VAN (*n* = 115)	Sleep disturbances + MVAD (*n* = 152)	Sleep disturbances + VAD (*n* = 415)	*P* value ^**a**^
**CSHQ total score, mean (SD)**	40.63 (2.58)	47.72 (2.99)	47.99 (3.47)	< 0.001^***^
**CARS score, % (n)**				
Mild to moderate degree (30–36)	32.17 (37/115)	0 (0/149)	0 (0/418)	0.001^***^
Severe degree (37–60)	67.83 (78/115)	100 (149/149)	100 (418/418)	
**ABC total score, mean (SD)**	67.87 (5.78)	106.92 (23.30)	105.66 (22.10)	< 0.001^***^
**SRS total score, mean (SD)**	99.64 (11.80)	152.53 (25.77)	148.63 (24.98)	< 0.001^***^

*Abbreviations*: *ASD* Autism spectrum disorder, *CSHQ* Childhood Sleep Habit Questionnaire, *CARS* Childhood Autism Rating Scale, *ABC* Autism Behavior Checklist, *SRS* Social Responsiveness Scale, *VAN* Vitamin A normal, *MVAD* Marginal vitamin A deficiency, *VAD* Vitamin A deficiency, *SD* Standard deviation

^***^P < 0.001

^a^VAD with MVAD and VAN was recognized as significant by Least Significant Difference (LSD)(*P* < 0.001)

In summary, although the children with ASD without sleep disturbances had higher VA levels than those with ASD with sleep disturbances, whose VA levels were comparable to the VA levels of TDC, individuals with ASD in general had lower VA levels and a higher prevalence of sleep disturbances than TDC. Results suggest that children with ASD with sleep disturbances had severely deficient VA levels.

### VA levels and sleep disturbances associated with autism symptoms

To determine the association between VA levels and sleep disturbances in children with ASD, we initially estimated the CARS, ABC, and SRS scores of children with ASD who had sleep disturbances or VAD. Results indicated that individuals with sleep disturbances had a higher score of core symptoms than those without sleep disturbances (i.e., higher CARS, ABC, and SRS scores) (Table 2). Furthermore, after stratifying the children with ASD with sleep disturbances by VA levels (VAN, MVAD, VAD), children in the VAD group had higher CARS, ABC, and SRS scores than those in the MVAD and VAN groups (Table 3).

Results of multivariable linear regression analyses performed sequentially demonstrated that VA levels in children with ASD had a significant negative relationship with sleep disturbances [B (standard error [SE]) = − 5.307 (1.234), 95% CI: − 6.295–-4.319, *P* < 0.001]. Sleep disturbances had a significant positive relationship with CARS scores [B (SE) = 0.159 (0.022), 95% CI: 0.115–0.203, *P* < 0.001] and SRS scores [B (SE) = 0.053 (0.008), 95% CI: 0.038–0.069, *P* < 0.001] (Table 4). We concluded that decreased VA levels were associated with an increase in sleep disturbances in children with ASD.

**Table 4:** Simple linear and multivariate regression analyses for the CSHQ total score of ASD children

Variables	Simple linear regression			Multivariable regression^a^		
	B (SE)	95% CI	*P* value	B (SE)	95% CI	*P* value
VA levels	−10.105 (0.395)	−10.882–-9.329	< 0.001^***^	−5.307 (1.234)	−6.295–-4.319	< 0.001^***^
CARS total score	0.42 (0.019)	0.384–0.458	< 0.001^***^	0.159 (0.022)	0.115–0.203	< 0.001^***^
ABC total score	0.11 (0.005)	0.094–0.116	< 0.001^***^	−0.018 (0.010)	−0.037–0.001	0.059
SRS total score	0.09 (0.004)	0.085–0.101	< 0.001^***^	0.053 (0.008)	0.038–0.069	< 0.005^**^

*Abbreviations*: *ASD*, Autism spectrum disorder, *CSHQ* Childhood Sleep Habit Questionnaire, *CI* Confidence interval, *VA* Vitamin A, *CARS* Childhood Autism Rating Scale, *ABC* Autism Behavior Checklist, *SRS* Social Responsiveness Scale

^**^P < 0.01, ^***^P < 0.001

^a^Multivariable regression model included all variables mentioned in the table. Beta estimates (standard errors) for continuous variables are shown

Based on the results above, to further investigate whether VA levels and sleep disturbances in children with ASD jointly affected autism symptoms, we performed two-way ANOVAs. Results showed that in the CARS evaluation, the main effects of VA levels (*P* < 0.01) and sleep disturbances (*P* < 0.01) were significantly related to the severity of autism symptoms (Fig. 2b, c). Importantly, VA levels and sleep disturbances interacted such that the greatest severity of ASD symptoms were in children with ASD who had both sleep disturbances and VAD (*P* < 0.001) (Fig. 2a). Similar ANOVAs were conducted for ABC and SRS scores, which revealed significant main effects of VA levels (*P* < 0.001) and sleep disturbances (*P* < 0.001) on both ABC and SRS scores in children with ASD (Fig. 2e, f, h, i); meanwhile, the interactions between VA levels and sleep disturbances were also significant and were associated with increased severity of core symptoms (as evaluated for the ABC and SRS scores) in children with ASD (Fig. 2d, g).

**Fig. 2:** The effect of VA levels and sleep disturbances on autism behaviors of children with ASD. **a** The effect of interaction between VA levels and sleep disturbances on CARS total score. **b** Independent effect of VA levels on the CARS total score. **c** Independent effect of CSHQ total score on CARS total score. **d** The effect of interaction between VA levels and sleep disturbances on ABC total score. **e** Independent effect of VA levels on ABC total score. **f** Independent effect of CSHQ total score on ABC total score. **g** The effect of interaction between VA levels and sleep disturbances on SRS total score. **h** Independent effect of VA levels on SRS total score. **i** Independent effect of CSHQ total score on SRS total score. The values are the means (standard deviation). ^**^P < 0.01, ^***^P < 0.001. VA, vitamin A; ASD, autism spectrum disorder; CARS, Childhood Autism Rating Scale; CSHQ, Childhood Sleep Habit Questionnaire; ABC, Autism Behavior Checklist; SRS, Social Responsiveness Scale; VAN, vitamin A normal; VAD, vitamin A deficiency

Collectively, we concluded that, in addition to reduced VA levels being associated with sleep disturbances among children with ASD, the interaction between VAD and sleep disturbances affected autism symptoms in children with ASD.

## Discussion

To the best of our knowledge, this is the first study to demonstrate in detail that VAD and sleep disturbances are closely associated with the core symptoms of ASD in a large cohort of children with ASD. First, we confirmed ours and others’ previous reports of VAD in children with ASD [24, 32, 33]. Second, VAD or sleep disturbances among children with ASD corresponded to the severity of autism symptoms in our study. Third, there was a correlation between the degree of VAD and the prevalence of sleep disturbances in children with ASD. Finally, and critically, there was a synergistic effect of VA levels and sleep disturbances, such that lower VA levels and increased sleep disturbances were associated with more severe autism symptoms in children with ASD.

Nutrient deficiencies, such as vitamin D, vitamin E, and calcium, commonly occur in children with ASD [34, 35]. A study evaluating the levels of vitamin D in adolescents revealed that poor quality sleep was associated with vitamin D deficiency [36]. Researchers also found that the children’s picky eating was related to sleep disturbances during development; however, if extra nutrients were supplied to mothers during lactation, the children were less prone to sleep disturbances [35]. Additionally, if extra nutrients were supplied to ASD children’s mothers during lactation, the children were less prone to sleep disturbances [37]. It is also worth noting that VA has been accepted as a necessary nutrient for regular patterns of brain activity and has been related to the development of ASD [38]. Additionally, we previously found that serum VA levels were positively correlated with language and social development in children [39].

In the present study, we investigated the influence of VA levels in children with ASD with sleep disturbances, confirming the prevalence of VAD in children with ASD and revealing the association between VAD and sleep disturbances in these children. Importantly, we determined the extent to which reduced VA levels and sleep disturbances negatively affected the core symptoms of children with ASD, providing preliminary data for further investigating the roles of VA in the pathogenesis and sleep disturbances during ASD. Consistent with our previous reports of gastrointestinal and sleep problems being related to behavioral symptoms in children with ASD [34], here we revealed that VA levels and sleep disturbances were associated with autism symptoms in children with ASD, indicating that nutrient deficiencies and behavioral comorbidities may work synergistically to facilitate ASD development. It is still unclear whether VAD and its correlation with sleep disturbances are specific to ASD. Nevertheless, based on our data, we conclude that VAD was closely related to sleep disturbances, and an interaction between VA levels and sleep disturbances was associated with the severity of autism symptoms in children with ASD. Moreover, our ongoing studies investigating molecular mechanisms in animal models have shown a role of VA in sleep via circadian rhythm regulatory genes (unpublished data). The role of VA in sleep physiology, particularly in circadian rhythms, has been reported by Sei [20]. As such, it is likely that VAD might be associated with sleep disturbances in ASD. Further study is required to elucidate this hypothesis.

In light of the prevalence of nutrient deficiencies in ASD, some researchers have conducted supplement interventions in children with ASD and found that children who took vitamin supplementation displayed considerable improvements in symptoms [39]. Indeed, we have previously shown that VA supplementation promoted changes in the gut microbiota composition, which had benefits regarding the improvement of autism [40] and relieving autistic symptoms [32]. We plan to continue this research and provide VA supplementation to children with ASD and VAD, and assess changes in autism symptoms and sleep disturbances in those individuals.

This study has a few limitations. First, this study was designed as a cross-sectional study; thus, causal inferences might be involved. Second, parts of the questionnaires were completed by the caregivers who all had different educational levels and attitudes, which might have contributed to some bias but did not affect the criteria for inclusion. Third, differences in lifestyles and customs, and the season of investigation might have had an indirect effect on our results in this study. Finally, the more determined relationship between VA levels, sleep disturbances, and core autism symptoms of children with ASD needs further elucidation.

## Conclusions

Children with ASD had lower serum VA levels and a higher prevalence of sleep disturbances. The degree of VAD was negatively correlated with the severity of sleep disturbances. Furthermore, the interaction between VA levels and sleep disturbances was associated with more severe autism symptoms in children with ASD.

## Data Availability

The datasets generated and/or analyzed during the current study are not publicly available because of another unpublished paper based on the data, but are available from the corresponding author on reasonable request.

## Abbreviations

ABC: Autism Behavior Checklist
ANOVA: Analysis of variance
ASD: Autism spectrum disorder
CARS: Childhood Autism Rating Scale
CI: Confidence interval
CSHQ: Childhood Sleep Habit Questionnaire
MVAD: Marginal vitamin A deficiency
SD: Standard deviation
SE: Standard error
SRS: Social Responsiveness Scale
TDC: Typically developing children
VA: Vitamin A
VAD: Vitamin A deficiency
VAN: Vitamin A normal
